The article "Multidimensional Information Network Big Data Mining Algorithm Relying on Finite Element Analysis" was published in 2022. Journal: Comput Intell Neurosci.

# Multidimensional Information Network Big Data Mining Algorithm Relying on Finite Element Analysis

**DOI:** 10.1155/2022/7156715

**Published:** 2022-04-11

**Authors:** Haifeng Li

**Affiliations:** Dalian Jiaotong University, Dalian, Liaoning 116028, China

## Abstract

In recent years, with the rapid development of the Internet, online social networks have been continuously integrated with traditional interpersonal networks and research on information dissemination in social networks has gradually increased. This article studies and analyzes the multidimensional information network big data mining algorithm based on the finite element analysis method. This paper firstly introduces the finite element analysis and calculation process, a finite element data mining simulation application software management system will integrate current data, calculation, and background data into one, then analyzes the data mining clustering algorithm, and conducts an experimental exploration of the influential node mining algorithm in complex networks. The experimental results show that the LIC algorithm is better than the CC algorithm, the DC algorithm, and the BC algorithm; its overall performance is improved by 30%, and the effect is better. The LIC algorithm can effectively and quickly determine the influential nodes, which is helpful for social network analysis.

## 1. Introduction

The important purpose of the research on the mining algorithm for the number of nodes with far-reaching influence in the social Internet is to excavate the number of *k* important nodes with far-reaching influence in the number of nodes in the entire social Internet and finally make these *k* nodes in an important position. Under this transfer mechanism, as many network nodes as possible are affected. In a word, the problem of important network nodes that are discovered from social networks and have a huge social influence also constitutes a problem of maximizing social influence to some extent. Among them, mining influential nodes in the network can inhibit or accelerate the dissemination and diffusion of information in the network. It takes the mined top-k nodes as a set of known seed nodes and finally maximizes the influence through a certain propagation strategy.

Due to the development of social Internet technology, the Internet has completely changed the way people communicate. Social networking on the Internet is recognized by more and more people, especially by young people, which directly results in the rapid expansion of the social Internet. The corresponding results are roughly as follows: First, the number of user groups in the social Internet is huge, and the interpersonal network established between user groups and user groups is becoming more and more complex; the update and change speed of community Internet information content is increasing, and the relationship between users and applications is also dynamic, which makes it more difficult to predict information content. Therefore, the research and development of social Internet-oriented data mining algorithms with the characteristics of efficiency and practical value has practicality and great scientific significance for solving real problems in the community. At the same time, the research on the mining algorithm and information dissemination model of influential nodes in social network has certain scientific research value and significance for real life.

According to the research progress at home and abroad, different scholars have also carried out certain cooperative researches in finite element analysis, multidimensional information network and big data mining inside the dormitory. Elliott and Thomas defined a new finite element method for numerical approximation of the solution of partial differential equations in the volume domain and surface partial differential equations lying on the boundary of the volume domain. The key idea is to perform a polyhedral approximation to the whole region containing the union of simplexes and to use piecewise polynomial boundary surfaces as the approximation of the surface [1]. Salonitis et al. proposes a new user-friendly optimization method for lattice component design for weight minimization, which combines finite element analysis and evolutionary calculations [2]. Li et al. analyzes the higher-order, central, finite-difference scheme of the diffusion equation in a finite interval. They analyzed stability through Gustafsson, Kreiss, and Sundström theories and eigenvalue visualization methods for semidiscrete and fully discrete schemes, followed by numerical tests to prove and validate the analytical results [3]. In order to retain important information related to mining of large data sets in multidimensional information networks, Xu presented an algorithm for constructing association rule mappings. On this basis, he proposed a multidimensional information network big data mining subalgorithm and an association rule generation algorithm, which were used for multidimensional information network big data mining and association rule generation, respectively. Finally, he demonstrated the feasibility and effectiveness of the algorithm through theoretical analysis and experimental comparison [4]. Wang proposed an indoor localization algorithm combining RSSI and nonmetric multidimensional scaling (NMDS) (RSSI-NMDS) to solve the problem that the indoor target localization algorithm based on received signal strength (RSSI) is susceptible to interference and large fluctuations in the Internet of Things environment [5]. Xu et al. takes a broader perspective on privacy issues related to data mining and studies various methods that help protect sensitive information. He identified four different types of users involved in data mining applications: data providers, data collectors, data miners, and decision makers [6]. However, these scholars did not rely on the finite element analysis method to study and analyze the multidimensional information network big data mining algorithm but only discussed its significance unilaterally.

The innovation of this article is as follows: (1) First, the finite element analysis calculation process is introduced. (2) The data mining clustering algorithm is analyzed, and the clustering analysis method refers to the analysis method of studying and processing the given object by means of computational mathematics. (3) Experimental analysis of the mining algorithm of influential nodes in complex networks is carried out.

## 2. Materials and Methods

A finite element data mining simulation uses a software management system that integrates current data, computing and background data. In the actual work of the finite element simulation analysis system, it first allows the user to use the software system to perform the preliminary data processing work of the finite element calculation with the help of the finite element data mining front-end. During this period, the structural model must be added first, and then the automatic mesh generation program is called directly to complete the setting of the finite element mesh pattern, and finally sets important technical parameters such as material properties through communication with users [7]. Finally, a scripted document of the initial data model can be obtained as input to the finite element calculation program. In the finite element calculation process, due to the deformation caused by the finite element meshing, after the finite element data mining is completed, the meshing program must be called to obtain the calculation data. Finally, after using the program, the user can perform an in-depth study and statistical analysis of the results of the finite element calculation process. In the entire finite element calculation process, the most important is the finite element solver. Other functional modules are used for the calculation of finite element solutions, but they are also an integral part of the system. Without any module, the system cannot work properly.  Figure 1 shows the service mode diagram of the finite element analysis and simulation system.

Although the finite element operation processing program is the most important part of the whole set of finite element analysis methods, the finite element operation processing program alone cannot provide an effective explanation for the actual project engineering. Therefore, on the one hand, the finite element calculation method involves many types of practical problems and a large amount of data and information. In the manual method to complete the data processing, the workload is large, the work efficiency is reduced, and errors are prone to occur; on the other hand, because the amount of information generated by the finite element operation is large and complicated, it is quite troublesome to analyze and use [8]. The finite element pre- and postprocessing software is a software technology that has flourished under this historical background.

Behavior is a series of purposeful, organized activities. There are usually two types: extrinsic behavior and intrinsic behavior. Learning behavior refers to the sum of activities that students undertake to achieve a certain learning effect under the guidance of a certain motivation. It is usually a series of activities in which students interact with their surroundings. Online learning behavior refers to the online learning that students conduct around certain learning goals, which can be set by themselves or designated by teachers. It is a collection of various explicit or implicit behaviors in learning activities. For example, uploading and downloading learning resources, learning courses on demand, publishing learning and troubleshooting, and communicating with other students [9, 10].

A large number of research results and applications in the field of data analysis and mining can be regarded as an important result of the natural evolution of technology. Strictly speaking, “data mining” usually refers to a broad concept in the industry, which should be more accurately called “mining knowledge from data” or “discovering knowledge from data”; the “data mining” in the strict sense is only a basic work stage in the entire scientific research workflow [11]. The general process of mining knowledge from data is shown in Figure 2.

The goal of data analysis and mining is to find meaningful or potential content from the information database. The main service functions are as follows:

1. Concept description: concept description can also be called data synthesis. Its main purpose is to extract and compress data, and then describe the complete information, or compare it with other objects. Summary Statistics gives a general overview of the statistics.
2. Analysis methods and predictions: classification methods and predictions are two completely different forms of statistical analysis data, which can be used to establish models to describe important statistical categories and to predict the future development of analysis methods [12]. In practical applications, classification prediction is widely used. For example, a classification model can be established to classify mobile users and return visits to high-frequency attrition groups as soon as possible to reduce user attrition; it is also possible to classify traffic flow information by establishing a classification model to predict future traffic congestion. Cluster analysis: The basic principle of cluster analysis is high cohesion and low mutual coupling. The final conclusion is that it has a high similarity to the same class of objects and a low similarity to other class objects [13].
3. Lonely point analysis: some objects in the database system may be different from the general behavior and model of data analysis, for this kind of object, we call it a lonely point. When people design data mining algorithms, they usually try to minimize the harm of lonely points, but in some special applications, the lonely point itself can also be an important judgment information. For example, in telecommunication spoofing checks, lonely spots can indicate spoofing activity [14].
4. Time series analysis: in time series analysis, the attribute values of data are constantly changing with time. These data are generally obtained at the same time interval but may be obtained at different time intervals. Data can be more visualized with time series plots.

Clustering refers to the process of distinguishing data signals according to specific conditions and rules. In this step, there is no prior knowledge of the relevant type, and there is no teacher's guidance, so it is in the scope of unsupervised classification.

Cluster analysis method refers to an analysis method that uses computational mathematics to study and process a given object. Clustering is an important and human act because a person's developmental process learns to recognize things by constantly reshaping subconscious aggregation patterns. The traditional cluster analysis method strictly defines various statistical objects to be aggregated, and the boundaries between classifications are very clear, so we can call it hard classification [15]. However, in general practical use, because most objects lack strict characteristic attribute definitions, and there is an unclear intermediary between the form and the class characteristic attributes, they have the characteristics of one and the other, so they are suitable for implementing soft classification.

### 2.1. Mathematical Model of Cluster Analysis

Supposing *A*={*a*_1_, *a*_2_,…, *a*_*m*_} is the whole object to be clustered (i.e. domain of discourse), among them, each object *a*_*i*_(1 ≤ *i* ≤ *m*) is called a sample, and the object is described by a plurality of parameter values, which represent a feature of the object. So each object *a*_*i*_ corresponds to a vector *V*(*a*_*i*_)=(*a*_*i*1_, *a*_*i*2_,…, *a*_*in*_), where *a*_*ij*_(1 ≤ *j* ≤ *n*) is the assignment of *a*_*i*_ on the jth feature and *V*(*a*_*i*_) is called the feature vector of *a*_*i*_ [16]. Cluster analysis is to analyze the spatial distance between the feature vectors corresponding to the samples in the universe A and their distribution and divide them into l disjoint pattern subsets according to the distance relationship between each sample and satisfy the following formula conditions:

(1) $$\begin{array}{c} A_{1}\cup^{}A_{2}\cup^{}\ldots \cup^{}A_{l}=A,\\ A_{i}\cap^{}A_{j}=\emptyset \;\left(1\leq i,j\leq l,i\neq j\right). \end{array}$$

Membership function *u*_*ij*_ represents the membership of sample *a*_*j*_(1 ≤ *j* ≤ *m*) with respect to subset (class) *A*_*j*_(1 ≤ *i* ≤ *l*), as follows:

(2) $$\begin{array}{c} u_{a_{i}}\left(a_{j}\right)=u_{ij}=\left\{\begin{array}{c} 1\left(a_{j}\in A_{i}\right),\\ 0\left(a_{i}\in A_{j}\right). \end{array}\right) \end{array}$$

As shown in the previous formula, the membership function must satisfy *u*_*ij*_ ∈ *N*_*sl*_, that is, each sample can only belong to one of the classes, and each subclass is required to be a nonempty set.

(3) $$\begin{array}{c} N_{sl}=\left\{u_{il}|u_{ij}\in \left\{0,1\right\},\overset{l}{\underset{i=1}{\sum }}u_{ij}=1,\forall j;0<\overset{m}{\underset{j=1}{\sum }}u_{ij}<m,\forall i\right\}. \end{array}$$

In the real world, the membership degree of a sample may not be either one or the other. From this, fuzzy theory is introduced, which becomes a fuzzy set class, and the sample set *A* is divided into multiple fuzzy subsets ${\tilde{A}}_{1},{\tilde{A}}_{2},\ldots ,{\tilde{A}}_{l}$, and the membership function *u*_*ij*_ of the sample is extended from the binary case of {0, 1} to the [0, 1] interval, satisfying the conditions:

(4) $$\begin{array}{c} \sup v\left({\tilde{A}}_{i}\right)=A,u_{ij}\in \left[0,1\right],\\ \overset{l}{\underset{i=1}{\sum }}u_{ij}=1\left(\forall j\right),0<\overset{m}{\underset{j=1}{\sum }}u_{ij}<n, \end{array}$$

where sup represents the support set of the fuzzy set.

### 2.2. Fuzzy Clustering Objective Function

Mathematical model based on cluster analysis, if fuzzy concept is introduced. It uses the membership degree *o*_*il*_ of the sample point *a*_*l*_ and the sample prototype of the *i*-th class as the weight to weight the distance. At this time, the objective function of the cluster analysis is given as follows:

(5) $$\begin{array}{c} J_{1}\left(O,V\right)=\overset{b}{\underset{i=1}{\sum }}\overset{m}{\underset{l=1}{\sum }}o_{il}{\left(h_{il}\right)}^{2},\;O\in R_{s}. \end{array}$$

After fuzzy clustering the objective function of the hard clustering analysis method, it uses the sum of squares of membership to transform the objective function of the sum of squares of errors into the objective function of all weighted sums of squares of errors, namely,

(6) $$\begin{array}{c} J_{2}\left(O,V\right)=\overset{b}{\underset{i=1}{\sum }}\overset{m}{\underset{l=1}{\sum }}o_{il}{}^{2}{\left(h_{il}\right)}^{2},\;O\in R_{s}. \end{array}$$

### 2.3. Objective Function of General Fuzzy Cluster Analysis

Among the more general expressions are

(7) $$\begin{array}{c} J_{n}\left(O,V\right)=\overset{b}{\underset{i=1}{\sum }}\overset{m}{\underset{l=1}{\sum }}o_{il}{}^{n}{\left(h_{il}\right)}^{2},\;O\in R_{s}, \end{array}$$

where *h*_*il*_ is a distance norm, and the distance *h*_*il*_ between the sample point *a*_*l*_ and the cluster center *v*_*i*_ of the *i*-th class represents the similarity between the sample point and the cluster center, which can generally be expressed as follows:

(8) $$\begin{array}{c} h_{il}{}^{2}=a_{l}-v_{iX}\\ ={\left(a_{l}-v_{i}\right)}^{Q}X\left(a_{l}-v_{i}\right), \end{array}$$

where *n* ∈ [1, *∞*) is the weighting index, also known as the smoothing parameter, which controls the fuzzy degree of fuzzy clustering. The larger the *n* is, the larger the blurring degree is; the smaller the *n* is, the smaller the blurring degree is [17]. Because *n* controls the degree to which membership is shared among classes, the larger *n*, the greater the ambiguity. After research, it is found that for different application scenarios, the optimal *n* can be in the range of 1 to 5, and *n* = 2 is usually selected.

### 2.4. Analysis and Solution Process Based on Objective Function Clustering Algorithm

In order to obtain the optimal solution of the objective function of fuzzy clustering, the criterion of clustering can be taken, that is, ∑_*i*=1_^*b*^*o*_*il*_=1 and min{*J*_*n*_(*O*, *V*)} are obtained under the constraints of the mechanism, namely,

(9) $$\begin{array}{c} \min\left\{J_{n}\left(O,V\right)\right\}=\min\left\{\overset{m}{\underset{l=1}{\sum }}\overset{l}{\underset{i=1}{\sum }}{\left(o_{il}\right)}^{n}{\left(h_{il}\right)}^{2}\right\}\\ =\overset{m}{\underset{l=1}{\sum }}\min\left\{\overset{b}{\underset{i=1}{\sum }}{\left(o_{il}\right)}^{n}{\left(h_{il}\right)}^{2}\right\}. \end{array}$$

Therefore, this problem can be understood as follows: under the condition of membership degree, ∑_*i*=1_^*b*^*o*_*il*_=1, obtain

(10) $$\begin{array}{c} \min\left\{\overset{b}{\underset{i=1}{\sum }}{\left(o_{il}\right)}^{n}{\left(h_{il}\right)}^{2}\right\}. \end{array}$$

Using Lagrange's theorem to solve, we can get the expression of the membership degree corresponding to the jth object:

(11) $$\begin{array}{c} o_{il}=\frac{1}{{\sum_{i=1}^{b}\left[h_{jl}/h_{il}\right]}^{2/n-1}}. \end{array}$$

The fuzzy classification matrix usually satisfies the following conditions:

1. *o*_*il*_ ∈ [0,1], that is, each element in the matrix is between 0 and 1 closed interval
2. ∑_*i*=1_^*b*^*o*_*il*_=1, the sum of the elements of each column is 1, that is, the sum of the membership degrees of each element to all classes is 1
3. ∑_*i*=1_^*b*^*o*_*il*_ > 0, this condition ensures that each class is not empty

Similarly, the cluster center of fuzzy clustering can be obtained as follows:

(12) $$\begin{array}{c} V_{i}=\frac{\sum_{l=1}^{m}{\left(o_{il}\right)}^{n}a_{l}}{\sum_{l=1}^{m}{\left(o_{il}\right)}^{n}}. \end{array}$$

It can be seen that the cluster center can be obtained from the membership degree. The purpose of cluster analysis is to discover the implicit grouping information in the data. In order to represent this accuracy well, the effectiveness of clustering needs to be analyzed. When evaluating clustering results, the optimal number of clusters is usually an important indicator of effectiveness [18, 19].

In the process of optimizing the objective function, people have tried many methods such as dynamic programming, but the large storage space and long running time limit its popularization and application. The most widely used in practice is the iterative optimization algorithm, which is easy to enter the extreme point of the local area, so it is more sensitive to initialization, and one of the important input parameters is the number of clusters *k*. Although the exact value of *k* may not be known, it is usually possible to approximate the value of *k* by evaluating the quality of the clustering results at different *k*. Given an ideal cluster index, such as average radius or diameter, as long as the number of an imaginary cluster is less than or greater than the actual number of clusters, the index will tend to rise very slowly [20]. However, when trying to acquire far fewer clusters than the true number, the index increases rapidly. A schematic diagram of the above idea is shown in Figure 3.

Among them, for the evaluation of fuzzy clustering, the separation coefficient is expressed as follows:

(13) $$\begin{array}{c} G\left(O,h\right)=\frac{1}{m}\overset{m}{\underset{i=1}{\sum }}\overset{h}{\underset{j=1}{\sum }}{\left(o_{ij}\right)}^{2}, \end{array}$$

where *o*_*ij*_ is the fuzzy membership degree of data object *i* belonging to cluster *j*, assuming all clustering results here, then the number of clusters *k* is given by the following formula:

(14) $$\begin{array}{c} \max\left\{\max\;G\left(O;h\right)\right\},h=2,3,\ldots ,m-1. \end{array}$$

Similarly, a variant of the separation coefficient can be obtained, the separation entropy index:

(15) $$\begin{array}{c} L\left(O,h\right)=-\frac{1}{m}\overset{m}{\underset{i=1}{\sum }}\overset{h}{\underset{j=1}{\sum }}o_{ij}\log\left(o_{ij}\right). \end{array}$$

The corresponding number of clusters is given as follows.

If *o*_*ij*_ is close to 0 or 1, the smaller the entropy value and the better the clustering result. If *o*_*ij*_ is close to 0.5, the clustering ambiguity is high, the entropy value is large, and the corresponding clustering result is not good. These two indicators are proposed for partition-based fuzzy clustering, which is sensitive to fuzzy factors [21].

In the fuzzy k-means algorithm, due to the introduction of ∑_*i*=1_^*b*^*o*_*ih*_=1, in the case that the sample set is not ideal, it can be assumed that there are several isolated points far away from the clustering center of each class. Because the isolated point itself actually belongs to a certain class, under the original constraints, it will have a large degree of membership to various types or be approximately equal to each type of membership degree. This situation will affect the correctness of the final clustering results [22]. To overcome this shortcoming, we can relax the constraint and change it to

(16) $$\begin{array}{c} \overset{b}{\underset{i=1}{\sum }}\overset{m}{\underset{h=1}{\sum }}o_{ih}=\beta ,\beta \in \left[1,m\right). \end{array}$$

That is, the sum of the membership degrees of all samples to each category is *β*, a positive integer value. At this time, on the premise of Formula (16), obtain min{*J*_*n*_(*O*, *V*)}, and the solution method is the same as above. At this point, the membership degree should be

(17) $$\begin{array}{c} o_{ih}=\beta \frac{1}{\sum_{i=1}^{b}\sum_{i=1}^{m}{\left[s_{jh}/s_{ih}\right]}^{2/n-1}}. \end{array}$$

Obviously, this condition is completely different from the membership function in the traditional sense, and the membership degree estimated by the improved fuzzy k-means algorithm may exceed 1. If necessary, the obtained membership value can be normalized, which will not affect the final clustering result under normal circumstances.

The improved method has better adaptability than the original algorithm. It can not only obtain better processing results for clustering in the case of special isolated points but also relax the constraints of membership degree. As a result, the original result is less sensitive to the predetermined number of clusters than the clustering result. When the number in the cluster analysis method determined in advance is much lower than the value of the theoretical number of clusters, the fuzzy k-means calculation using this method can obtain a more accurate cluster analysis method center result.

However, if a certain cluster center is very close to a certain sample in the iterative process, then a cluster containing only one sample may be obtained in the end. To prevent this from happening, a nonlinear process can be added to the distance operation in *o*_*ih*_, so that the minimum calculated distance is not less than a certain threshold.

The usual distance measure in classical k-means clustering algorithm and fuzzy k-means clustering algorithm adopts Euclidean distance or Manhattan distance. The Kowski distance is a generalization of these two distances, and it is defined as follows:

(18) $$\begin{array}{c} s\left(i,j\right)={\left({\left|a_{i1}-a_{j1}\right|}^{t}+{\left|a_{i2}-a_{j2}\right|}^{t}+\ldots +{\left|a_{iv}-jv\right|}^{t}\right)}^{1/t}. \end{array}$$

When *t* = 1, it is the Manhattan distance, and when *t* = 2, it means the Euclidean distance.

In cluster analysis, often fields in a data set may maintain an established or obvious weighting relationship. For example, in the cluster analysis of mobile customers, the age, income, and other classification weights of customers are significantly larger, while the weight of noise points is significantly smaller. So, we get the weighted Euclidean distance:

(19) $$\begin{array}{c} s\left(i,j\right)={\left(u_{1}{\left|a_{i1}-a_{j1}\right|}^{2}+u_{2}{\left|a_{i2}-a_{j2}\right|}^{2}+\ldots +u_{v}{\left|a_{iv}-jv\right|}^{2}\right)}^{1/2}. \end{array}$$

The advantage of this method is that it can find more accurate cluster centers than the original algorithm, the disadvantage is that it is difficult to determine the size of the weights. In order to realize the automation and intelligence of weight judgment, it can consider weighting each sample through the improved membership function. The weights of noise samples after relaxing the membership constraints are usually small, so the expected purpose is achieved. Then, the minimum value of the objective function is obtained to realize cluster analysis.  Figure 4 shows the cluster analysis process.

## 3. Results and Analysis

### 3.1. Influential Node Mining Algorithm for Complex Networks

The evaluation of the influence of nodes in complex networks can make information spread faster and more widely, which is of great significance in practical applications. According to the characteristics of complex networks, this article proposes a Local Importance Centrality Algorithm (LIC), which is a new method for evaluating the influence of nodes in complex networks based on network local characteristics, such as degree and clustering coefficient. The local importance centrality algorithm can more effectively identify influential nodes.

### 3.2. Experimental Data Set

The data sets used in this experiment are collected from real networks: Netscience, E-mail, and Power.

Netscience data set publishes a topological graph of collaborations between authors of articles on topic networks, in which scientists represent nodes and collaborations represent edges. The data set contains a total of 1589 scientists, using the largest subgraph with 379 nodes in it. The basic data parameters of the data set are shown in Table 1.

E-mail data set represents the topology of e-mail forwarding relationships among Rovira University members, where Rovira University members represent nodes and forwarding relationships between members represent edges. The data parameters are shown in Table 2.

Power data set contains an undirected and unweighted topology map of the National Grid in the western United States. Nodes represent transformers, substations, and generators, and the relationship is a high-voltage transmission line. The basic data parameters of the network are shown in Table 3.

### 3.3. Experimental Results and Analysis

#### 3.3.1. Relationship between the Rank Evaluated by Various Centrality Algorithms and the Average Influence Value < *F*(*t*) >

In this article, the SIR infectious disease model is used to simulate the propagation on three real network data sets, and the top-rank of the influence ranking obtained by the DC algorithm, the BC algorithm, the CC algorithm, and the LIC algorithm is compared experimentally.

Only one node is selected as the initial infection node for each execution of influence propagation, and other nodes are susceptible nodes. Then, the information or virus spreads according to the mechanism of the SIR infectious disease model. After *n* executions (each node has one and only one initial infection node), the correlation between the node influence value *F*(*t*) and the four centrality algorithms can be examined. In order to further clarify the performance of several centrality algorithms, calculate the average influence value <*F*(*t*)> of the top-k nodes of each algorithm, where <*F*(*t*)> is the average of all *F*(*t*)s after *n* executions.

Comparisons are made on the Netscience data set. As shown in Figure 5, if the propagation performance of the centrality algorithm is good, then the top-k ranking Rank and <*F*(*t*)> should be negatively correlated, and the curve is downward sloping. That is, as the Rank increases, the nodes can influence (infect) fewer nodes.

Figure 6 shows the curves of the four algorithms are all downward sloping, and the curve of the degree centrality algorithm (DC) fluctuates greatly, which shows that the Rank calculated by the DC algorithm is quite different from the actual influence value. The curve of the DC algorithm is at the bottom of the four curves, which further shows that the top-k nodes discharged by the DC algorithm have a relatively low influence. The betweenness centrality algorithm (BC) also has a large curve and performs worse than the closeness centrality algorithm (CC) and the locally important centrality algorithm (LIC). The performance of the LIC algorithm is slightly better than that of the CC algorithm, and the two curves are relatively close.

On the E-mail data set, Figure 6 shows that the experimental results of the four centrality algorithms in this data set are all good. The top-k nodes sorted by the four algorithms can affect many nodes. It can be seen that the effect of the LIC algorithm is the best among the four centrality algorithms, and its curve fluctuation is relatively smooth. The effect of the CC algorithm in the figure is also very good. The <*F*(*t*)> of the BC algorithm and the DC algorithm are very high, but the curve fluctuations of the two are relatively large and the correlation is poor.

#### 3.3.2. Comparison of the Influence of Top 10 Nodes Based on the Sorting of Several Centrality Algorithms

In this round of experiments, the random sorting algorithm was added for comparison. This article compress the influence *F*(*t*) of different nodes in the top-10 node list evaluated by these five algorithms. Because the same nodes in the top-10 list are excluded, the performance of each algorithm can be compared better. Figures 7 and 8 show that on the Netscience data set, the LIC algorithm is compared with the BC algorithm, the CC algorithm, the DC algorithm, and the random algorithm. The total number of infected and immune nodes increases with time *t* and eventually reaches a stable value. It can be seen that although the convergence speed of the LIC algorithm is slightly lower than that of the CC algorithm and the DC algorithm, it can infect more nodes than the two algorithms. The LIC algorithm can obviously infect more nodes than the Random algorithm.

Figure 9 shows the comparison of the influence *F*(*t*) of the LIC algorithm and the DC algorithm at time *t* on the E-mail data set and the Power data set, respectively. The convergence speed of the LIC algorithm is significantly higher than that of the DC algorithm.

In Table 4, the average *F*(*t*) value of the top-10 nodes of the four algorithms is calculated. It can be seen that the average value of *F*(*t*) of the LIC algorithm is slightly better than that of the CC algorithm, its performance is improved by 30%, and the effect is better, and both are better than the DC algorithm and the BC algorithm.

This article proposes a new centrality algorithm based on network local importance for mining the influence of nodes in social networks. To verify the effectiveness and superiority of the algorithm, it uses the SIR infectious disease model to simulate the actual spreading influence of sorted list nodes evaluated by different centrality algorithms. The experimental results on three real social network data sets show that the influence nodes mined by the local importance centrality algorithm (LIC) are significantly better than the betweenness centrality algorithm (BC) and the degree centrality algorithm (DC). The influence effect is close to the closeness centrality algorithm (CC) and is much lower than the closeness centrality algorithm (CC) in computational time complexity. This shows that the LIC algorithm can solve the shortcomings and deficiencies of the existing centrality algorithms and can effectively and quickly determine the influential nodes, which is helpful for social network analysis and has important practical significance.

## 4. Discussion

The current research results show that some network nodes in social portals have great social influence, which can promote or limit the dissemination of information to a certain extent. These network nodes reduce the energy consumption of traditional Internet computing resources to a certain extent and give full play to the function of effectively optimizing traditional Internet information resources. Therefore, finding and classifying influential network nodes has become an urgent problem for many experts and scholars. The characteristic of the social network analysis method compared with the other two methods is to analyze the network characteristics without destroying the network structure. This method is universal and suitable for most social networks. The social network analysis method mainly relies on analyzing the basic topological characteristics of the network, such as the degree of the node, the shortest path, the eigenvector, and other indicators to evaluate the influence of the node.

## 5. Conclusion

In this article, the influence of nodes is approximated by the local importance of nodes in the network, and a new algorithm based on the local importance centrality of the network (LIC algorithm) is proposed. The local importance of nodes is calculated and evaluated according to local information such as network moderateness and aggregation coefficient, so the computational time complexity is relatively low. By comparing it with the degree centrality algorithm (DC), the betweenness centrality algorithm (BC) and the closeness centrality algorithm (CC), it proves that it has a high influence correlation with the local important centrality algorithm, so that important influential nodes can be well mined. In this article, the research on mining key nodes in the social Internet is mainly based on the current more common way to evaluate the influence of nodes through node centrality. But in real, online, social networking sites, users' influence is not only evaluated by topological characteristics among users, but some more personalized characteristics, such as user attributes, preferences, and the like. Therefore, the next research work is to add attributes such as user personalization characteristics on the basis of complex network topology characteristics to evaluate user influence.

## Figures and Tables

**Figure 1:** Service mode diagram of the finite element analysis simulation system.

**Figure 2:** The whole process of knowledge discovery in data.

**Figure 3:** Trend diagram of the number of *k* versus the average diameter of clusters.

**Figure 4:** Cluster analysis.

**Figure 5:** Comparison of the correlation between Rank and <*F*(*t*)> on the Netscience data set.

**Figure 6:** Correlation comparison between Rank and <*F*(*t*)> on the E-mail data set.

**Figure 7:** Comparison of the number of infected nodes between the LIC algorithm and other algorithms in time *t* (1).

**Figure 8:** Comparison of the number of infected nodes between the LIC algorithm and other algorithms in time *t* (2).

**Figure 9:** Comparison of the influence *F*(t) between the LIC algorithm and the DC algorithm at time *t*.

**Table 1:** Basic network parameters of the Netscience data set.

Statistical item	Statistics	Statistical item	Statistics
Number of nodes (*n*)	381	Maximum degrees	36
Number of sides (*m*)	916	Clustering coefficient	0.39
Average degrees	4.79	Average shortest distance	5.98

**Table 2:** Basic network parameters of E-mail data set.

Statistical item	Statistics	Statistical item	Statistics
Number of nodes (*n*)	1098	Maximum degrees	69
Number of sides (*m*)	5469	Clustering coefficient	0.13
Average degrees	9.57	Average shortest distance	3.697

**Table 3:** Basic network parameters of the Power data set.

Statistical item	Statistics	Statistical item	Statistics
Number of nodes (*n*)	5021	Maximum degrees	20
Number of sides (*m*)	6603	Clustering coefficient	0.13
Average degrees	2.58	Average shortest distance	19.02

**Table 4:** Average <*F*(*t*)> values of top 10 nodes for each centrality algorithm.

Data set	LIC	DC	BC	CC
Netscience	359.8	358.7	357.3	358.3
E-mail	1009.8	996.2	1005.5	1010
Power	1399.6	589.1	1389.7	1393.2

## Data Availability

The data used to support the findings of this study are available from the author upon request.
